# Trophinin Is an Important Biomarker and Prognostic Factor in Osteosarcoma: Data Mining from Oncomine and the Cancer Genome Atlas Databases

This article has been retracted.

**DOI:** 10.1155/2021/6885897

**Published:** 2021-07-06

**Authors:** Pan Cai, Yan Lu, Zhifeng Yin, Xiuhui Wang, Xiaoxiao Zhou, Zhuokai Li

**Affiliations:** ^1^Department of Orthopedics, Zhoupu Hospital, Affiliated to Shanghai University of Medicine & Health Sciences, Shanghai 201318, China; ^2^Department of Laboratory Medicine, Zhoupu Hospital, Affiliated to Shanghai University of Medicine & Health Sciences, Shanghai 201318, China; ^3^Department of Orthopedics, Shanghai Zhongye Hospital, 200941 Shanghai, China

## Abstract

Osteosarcoma (OS) is a type of bone malignancy with a high rate of treatment failure. To date, few evident biomarkers for the prognostic significance of OS have been established. Oncomine was used to integrate RNA and DNA-seq data from the Gene Expression Omnibus (GEO), The Cancer Genome Atlas (TCGA), and the published literature. The correlation of the gene Trophinin (TRO) and different types of cancers was generated using the Cancer Cell Line Encyclopedia (CCLE) online tool. Prognostic values of featured Melanoma Antigen Gene (MAGE) members were further assessed by establishing the overall survival using the Kaplan-Meier plotter. Moreover, the online tool, Database for Annotation, Visualization and Integrated Discovery version (DAVID), was used to understand the biological meaning list of the genes. MAGEB10, MAGED2, TRO, MAGEH1, MAGEB18, MAGEB6, MAGEB4, MAGEB1, MAGED4B, MAGED1, MAGEB2, and MAGEB3 were significantly overexpressed in sarcoma. TRO was further demonstrated to be distinctively upregulated in osteosarcoma cell lines and associated with shorter overall survival. TRO may play an important role in the development of OS and may be a promising potential biomarker and prognostic factor.

## 1. Introduction

Osteosarcoma (OS) is the most common bone malignancy in young people, with over 50% of cases occurring in the first two decades of life [1]. Tremendous progress has been achieved in the past few decades in the field of OS therapy development including advances in surgical and diagnostic strategies and the use of combined chemotherapy [2]. Despite this progress, curative treatment of OS remains challenging with subsequent poor prognosis and shortened life expectancy [3]. Early diagnosis and treatment of OS, particularly with nonmetastatic OS, is crucial for improving the prognosis of OS patients [4]. Unfortunately, few distinctive diagnostic and prognostic biomarkers have been identified. A better understanding of the molecular and cellular biology and an identification of effective biomarkers involved in tumor initiation and progression are crucial for optimizing diagnosis and treatment of OS.

The TRO gene encodes for Trophinin, a member of the Melanoma Antigen Gene (MAGE) family, mediate the initial attachment of the blastocyst to the uterine epithelial cells during embryo implantation through a cell adhesion molecule complex in combination with bystin and tastin [5]. Furthermore, a prior study indicated that TRO is overexpressed in many trophoblastic cancers, which is of great importance for the progression of trophinin-expressing cancers [6]. TRO may therefore have a critical role in the development of different cancers, with a possible role in OS initiation and prognosis remaining elusive.

In the present research, we first investigated the diagnostic role and prognostic value of TRO in OS. Additionally, the underlying biological mechanism of TRO in OS was explored.

## 2. Materials and Methods

### 2.1. Oncomine Analysis

The Oncomine (https://www.oncomine.org) database integrates RNA and DNA-seq data from GEO, TCGA, and published literature. We can use Oncomine for differentially expressed gene analysis, clinical correlation analysis, and multigene coexpression analysis. The expression information of the MAGE family in sarcoma and coexpressed genes of the MAGE family were retrieved from Oncomine with the default setting of fold change > 2 and *P* value < 0.01.

### 2.2. CCLE Analysis

The CCLE database (https://portals.broadinstitute.org/ccle/home) is an online encyclopedia of a compilation of gene expression, chromosomal copy number, and massively parallel sequencing data from 1457 human cancer cell lines and 136,488 unique data sets, to facilitate the identification of genetic, lineage, and predictors of drug sensitivity. The correlation of gene TRO and different types of cancers was generated using the CCLE online tool.

### 2.3. The Kaplan-Meier Plotter Survival Analysis

The MAGE members that were shown to be specifically highly expressed in sarcoma samples and their coexpressed genes were further assessed by displaying the overall survival using the Kaplan-Meier plotter (http://kmplot.com/analysis/). The Kaplan-Meier plotter is an online tool applied to assess the effect of 54,675 genes on survival using 13,316 cancer samples in 21 cancer types. Sources for the databases include GEO, EGA, and TCGA. The primary purpose of the tool is a meta-analysis-based discovery and validation of survival biomarkers. *P* < 0.01 was considered to indicate a statistically significant result.

### 2.4. Gene Ontology (GO) and Kyoto Encyclopedia of Genes and Genomes (KEGG) Pathway Enrichment Analysis

The online tool Database for Annotation, Visualization and Integrated Discovery version (DAVID) Bioinformatics Resources 6.8 was used to understand the biological meaning of the list of genes. GO enrichment and KEGG pathway analyses were performed with DAVID. The GO and KEGG pathway analysis result was visualized by the ggPlot2 R package. The relationship between GO terms was calculated in Cytoscape 3.7.2, using the plug-in software ClueGO.

## 3. Results and Discussion

### 3.1. Oncomine Analysis

Oncomine analysis revealed that for MAGE family, MAGEB10, MAGED2, TRO, MAGEH1, MAGEB18, MAGEB6, MAGEB4, MAGEB1, MAGED4B, MAGED1, MAGEB2, and MAGEB3 were significantly overexpressed in sarcoma, based on the TCGA database (Figure 1). The meta-analysis combined 27 studies ranking the MAGE family genes expressed in sarcoma by *P* value and median. TRO was the top gene which was significantly upregulated in sarcoma (Figure 2). The coexpressed genes of TRO were identified using the coexpression online tool in Oncomine. The top ten genes were PTK7, ZNF135, ZC4H2, DZIP1, EPHB3, SMARCA1, MYH10, GPC, TSPYL5, and H2AFY2 (Figure 3).

### 3.2. CCLE Analysis

CCLE analysis agreed with the Oncomine results demonstrating that TRO was distinctively upregulated in the osteosarcoma cell lines (Figure 4(a)). In addition, the DNA copy number was relatively high in osteosarcoma (Figure 4(b)). Moreover, the Achilles shRNA knockdown results showed osteosarcoma was ranked second when ordered by dependency probability with TRO (Figure 4(c)).

### 3.3. The Kaplan-Meier Plotter Survival Analysis

For the top 10 MAGE family genes of TRO, MAGED4B, MAGED2, MAGED1, MAGEA5, MAGEF1, and MAGEA3 were associated with shorter overall survival (*P* < 0.05) (Figure 5). For the top 10 coexpressed genes of TRO, PTK7, ZNF135, DZIP1, EPHB3, SMARCA1, GPC4, and TSPYL5 were associated with shorter overall survival (*P* < 0.05) (Figure 6).

### 3.4. Gene Ontology (GO) and Kyoto Encyclopedia of Genes and Genomes (KEGG) Pathway Enrichment Analysis

The MAGE family and coexpressed genes were significantly enriched in the biological progress of nervous system development, cochlea morphogenesis, and positive regulation of mesenchymal cell proliferation; in cellular components of coreceptor activity involved in the Wnt signaling pathway, protein binding, and transmembrane-ephrin receptor activity; in molecular functions of integral component of plasma membrane, synapse, and intrinsic component of plasma membrane; in KEGG pathways of Wnt signaling pathway, axon guidance pathways, and signaling pathways regulating pluripotency of stem cells (Figure 7 and Table 1).

## 4. Discussion

OS is the most common type of bone malignancy with a high incidence in teenagers [7]. Early diagnosis and effective treatment of OS could remarkably decrease the high OS-related mortality [8, 9]. However, current therapies for advanced OS remain poor due to the lack of specific molecular targets. In this study, we first aimed to investigate the diagnostic role and prognostic value of TRO in OS.

TRO is a member of MAGE family members of which have previously been reported as effective targets for cancer immunotherapy [10]. TRO is a type of adhesion molecule with specific expression on human trophoblast cells [11]. Trophoblastic cancer patients with high expression of this molecule often have poor prognosis [12]. Among those with positive expression of TRO, HMGB1/RAGE are often coexpressed, suggesting that TRO can promote tumor invasion through an HMGB1/RAGE signaling pathway [13]. Similarly, high levels of TRO were found to be related with poor prognosis in liver and gallbladder cancer [14, 15]. It has also been demonstrated that TRO enhanced invasion and promoted colorectal cancer through a mechanism involving HMGB1/RAGE [11]. However, the function of TRO in the prognosis and progression of OS had not yet been fully elucidated.

This study first investigated the function and clinical significance of TRO in OS patients via the clinical data of OS patients and public expression profiles. The results indicated that the members of the MAGE family, including MAGEB10, MAGED2, TRO, MAGEH1, MAGEB18, MAGEB6, MAGEB4, MAGEB1, MAGED4B, MAGED1, MAGEB2, and MAGEB3, were significantly overexpressed in sarcoma tissues. And TRO was further demonstrated to be distinctively upregulated in OS cell lines and associated with shorter overall survival. Moreover, it was indicated from the statistical analysis that there was an evident correlation between TRO expression levels and a relatively poor prognosis. It was verified by further univariate and multivariate analyses that TRO could be used as a potential prognostic biomarker for OS patients.

To the best of our knowledge, the regulation of the expression of TRO in OS patients has not yet been explored. A limited number of studies have reported that overexpression of other MAGE family numbers, such as melanoma antigen family A (MAGEA), and preferentially expressed antigen in melanoma (PRAME) are related to OS progression [16]. However, the specific mechanism of MAGE family contribution to the occurrence, development, and prognosis of OS is still unknown. The present study suggested that TRO can act as a promising biomarker for OS diagnosis and prognosis. Nevertheless, the current study presented results derived solely from bioinformatics analyses, and further experimental evidence is required to validate these findings.

## 5. Conclusions

Overall, as TRO is overexpressed in human OS tissues, a poor prognosis can be predicted by a high level of TRO. Therefore, our findings highlight that TRO may be an important biomarker for the prognosis and progression of OS.

## Figures and Tables

**Figure 1:** 

**Figure 2:** 

**Figure 3:** 

**Figure 4:** 

**Figure 5:** 

**Figure 6:** 

**Figure 7:** 

**Table 1a:** (a) Biological processes

Term	Name	Count	P-value	Genes
GO:0007399	Nervous system development	9	2.22E-6	SEMA6A, EFNB3, DPYSL4, MDK, ZC4H2, PCDHB3, APBA2, PAFAH1B3, GPM6B
GO:0090103	Cochlea morphogenesis	4	3.90E-5	FZD2, PTK7, WNT5A, SOX9
GO:0002053	Positive regulation of mesenchymal cell proliferation	4	6.53E-5	WNT5A, LRP5, SOX9, FGFR2

**Table 1b:** (b) Molecular functions

Term	Name	Count	P-value	Genes
GO:1904929	Coreceptor activity involved in Wnt signaling pathway	2	1.83E-2	PTK7, GPC4
GO:0005515	Protein binding	36	1.85E-2	ISYNA1, MAGED1, ZC4H2, MAGEF1, LRP5, EFNA4, MAGEA9, TRO, CCND2, DPYSL4, SOX9, GPRASP1, MYH10, MAGEA3, TLE2, SEMA6A, FZD2, TLE1, CADM1, IGFBP2, WNT5A, LDOC1, SMARCA1, TBX3, PTK7, ADGRL1, ZNF415, MAGED2, BCOR, DZIP1, APBA2, ZNF334, PAFAH1B3, FGFR2, TSPYL5, ITM2C
GO:0005005	Transmembrane-ephrin receptor activity	2	2.74E-2	EFNB3, EFNA4

**Table 1c:** (c) Cellular components

Term	Name	Count	P-value	Genes
GO:0005887	Integral component of plasma membrane	11	2.19E-2	TRO, SEMA6A, EFNB3, CADM1, TUSC3, PTK7, PCDHB3, GPC4, EFNA4, FGFR2, EPHB3
GO:0045202	Synapse	7	2.53E-2	CADM1, ZC4H2, COL4A5, ADGRL1, APBA2, MYH10, FGFR2
GO:0031226	Intrinsic component of plasma membrane	11	2.82E-2	TRO, SEMA6A, EFNB3, CADM1, TUSC3, PTK7, PCDHB3, GPC4, EFNA4, FGFR2, EPHB3

**Table 1d:** (d) KEGG pathways

Term	Name	Count	P-value	Genes
hsa04310	Wnt signaling pathway	4	7.12E-4	FZD2, CCND2, WNT5A, LRP5, GPC4
hsa04360	Axon guidance	4	6.41E-3	SEMA6A, EFNB3, EFNA4, EPHB3
hsa04550	Signaling pathways regulating pluripotency of stem cells	4	8.39E-3	FZD2, WNT5A, FGFR2, TBX3

## Data Availability

The data used to support the findings of this study are available from the corresponding author upon request.
